The article "Design-Centered HRI Governance for Healthcare Robots" was published in 2022. Journal: J Healthc Eng.

# Design-Centered HRI Governance for Healthcare Robots

**DOI:** 10.1155/2022/3935316

**Published:** 2022-01-07

**Authors:** Yueh-Hsuan Weng, Yasuhisa Hirata

**Affiliations:** ^1^FRIS, Tohoku University, Sendai, Japan; ^2^Department of Robotics, Tohoku University, Sendai, Japan

## Abstract

Recent developments have shown that not only are AI and robotics growing more sophisticated, but also these fields are evolving together. The applications that emerge from this trend will break current limitations and ensure that robotic decision making and functionality are more autonomous, connected, and interactive in a way which will support people in their daily lives. However, in areas such as healthcare robotics, legal and ethical concerns will arise as increasingly advanced intelligence functions are incorporated into robotic systems. Using a case study, this paper proposes a unique design-centered approach which tackles the issue of data protection and privacy risk in human-robot interaction.

## 1. Introduction

AI has great potential to support humans in their daily affairs and particularly in areas such learning and decision making. Nevertheless, with the advances in robotics, we are also going to see AI functions extend into physical environments. What is happening now is an emerging trend of coevolution of AI and robotics. The recently established Moonshot Research and Development Program in Japan mentions this trend in one of its strategic goals: “realization of AI robots that autonomously learn, adapt to their environment, evolve in intelligence and act alongside human beings, by 2050.” Under the goal, four types of next-generation AI robots for intelligent rescue, scientific discovery, interactive healthcare, and daily service have been selected for development. In the field of healthcare, the coevolution of AI will allow healthcare robots to become more integrated into the real world and provide sophisticated services to people. For example, developments could see robots that read patient's emotions and provide proper responses to them. Along this line, one of the more optimistic future scenarios is that advanced cognitive robots could enhance human users' self-efficacy through their comprehensive perception of the user's psychological states. In addition, this will demand a specific inter-platform design called “AI Robots Group,” which not only supports efficient circulation of user data for robot decision making, but also liberates robots from their hardware limitations. In other words, robots will not have a specific shape. They can change their physical bodies based on their tasks and service environments. Although the AI Robots Group enhances the adaptability of intelligent agents in human-robot interaction (HRI) to humans, it also raises many concerns in regard to ethics, law, and social implications regarding their design, release, and use.

The article "Design-Centered HRI Governance for Healthcare Robots" was published in 2022. Journal: J Healthc Eng.

Similar examples of previous discussions on privacy and data protection can be found in “Cloud Robotics” or “Networked Robotics.” Fosch-Villaronga and Millard mentioned the challenge of attributing legal responsibility in complex multiparty ecosystems [1], Pagallo has argued that when robots are more connected via the Internet, their interactive behaviors could cause harm in regard to “robotic privacy” [2]. Ishii has pointed out that the unpredictability of AI can cause new challenge for data protection, especially with regard to an algorithmic black box [3]. Taylor has proposed the necessity of considering a new level of data protection in data-driven emerging technologies. This has been labeled “group privacy” [4]. Indeed, the coevolution of technological trends in AI and robots will bring about many critical challenges to current data governance structures. First of all, current existing laws will become more ineffective in properly responding to risks of AI-driven emerging technologies. On the flip side, we must also avoid the overregulation of new technologies as it may hamper their development. This is something that happened in the 19^th^ century with the “Red Flag Laws” in the UK following the invention of steam powered vehicles [5]. This is also called the “pacing problem” [6]. However, as Oxford philosopher Bostrom has argued, once Artificial Narrow Intelligence agents break through the singularity and became Artificial General Intelligence entity, the next wave evolution towards a superintelligent entity can happen in a short period of time. In this case, regulators will not be able to have enough time to take a gradual process to improve the insufficient parts of current legislation due to the existential risks from a superintelligent entity [7]. Finally, the design objectives for AI-driven autonomous systems are not limited to mobility and functionality but also include “sociability.” Designers of socially intelligent machines will need to consider Value-Sensitive Design in order to make sure these machines serve human-centric principle [8]. Overall, the governance for autonomous systems will need to utilize design thinking and strategies to cover the gap between the advancement of systems and the inflexibility of regulatory norms.

## 2. Design-Centered Governance for Autonomous Systems

With the recent rise of AI technology and the accompanying increase in concern around the risks of AI, the concept of “Responsible AI by Design” has been widely adopted in many major ethical AI guidelines. For example, there is a central team at Google which conducts ethical reviews to ensure that their ongoing product projects are aligned with the company's AI principles which emphasize social benefit, safety, and accountability [9]. On the other hand, issues around a responsible design approach for AI governance at the level of human-robot interaction are relatively novel compared to what has been addressed in design practices in regard to algorithmic fairness, accountability, and transparency.

The article "Design-Centered HRI Governance for Healthcare Robots" was published in 2022. Journal: J Healthc Eng.

In terms of previous studies of ethical design approaches for AI governance in human-robot interaction, Cheon and Su used Value-Sensitive Design to analyze a collection of scientists' interviews from the IEEE database. They then integrated their digested ethical values stated in these interviews into a design framework for humanoid robots [10]. Wynsberghe has proposed the Care-Centered Value-Sensitive Design (CCVSD) as a framework for the ethical evaluation of care robots, so that design factors that have ethical concerns (i.e., use contexts, care practice, involved actors, etc.) can be clearlys presented as a reference for designers [11]. In addition to the top-down discussions on defining the framework and analyzing ethical values, another bottom-up challenge comes from the engineering side, which refers to problems we face when we apply ethical design in practice. Peters et al. have pointed out the difficulty for professional designers in directly applying ethical values from guidelines to design process. They also claim the importance of considering “process” rather than “framework” for ethical design [12]. Along this line of thought, in this paper we would like to propose a conceptual framework of Design-Centered Governance for Autonomous Systems which aims to address the above-mentioned problems via two design-centered approaches.

The first approach we need to consider is called “Ethically Aligned Design,” and we will look at how to embed ethical values in the design process of autonomous systems. Its purpose is to make sure that the decision making of autonomous systems can be aligned with human ethical standards. The IEEE Global Initiative on Ethics of Autonomous and Intelligent Systems is the world's primary organization for advocating the Ethically Aligned Design approach. In addition to wanting to ease people's fear of AI technology, they also want to prove that embedding ethical values in the design process of autonomous systems would be beneficial to technological innovation. In comparison to traditional approaches to repairment and punishment, this “Responsible AI by Design” is a way to bring about effective AI governance.

The article "Design-Centered HRI Governance for Healthcare Robots" was published in 2022. Journal: J Healthc Eng.

The approach of Ethically Aligned Design is not the same as ergonomics or industrial product design which focus on user demands. It is about design for values or a design method for ensuring that intelligent systems are aligned with human-centered moral values when they perform their tasks in human environments. In the future, we can expect more and more AI applications to be introduced into our daily life. It will be inefficient for these machines to perform their tasks if we only authorize a limited degree of autonomy in advance. In modern society, we have already used a Value-Sensitive Design approach to ensure that legal and ethical values can be protected by embedding certain functions inside technology products. “Technological Protection Measures” and “Privacy by Design” are two examples of using a Value-Sensitive Design approach to protect copyrights and data. Ethically Aligned Design can be seen as an extension of Value-Sensitive Design, but it has a special focus on design issues in intelligent and autonomous systems.

Regarding Ethically Aligned Design for human-robot interaction, there are previous related studies on machine ethics or “ethical protocol for HRI,” such as Ronald C. Arkin's Embedded Ethics architecture for military robots accessing the Laws of War (LOW) and Rules of Engagement (ROE) and Michal and Susan Leigh Anderson's MedEthEx: a prototype medical ethics advisor for supporting care robots to follow their prima facie duties in healthcare. However, these machine ethics projects have their limitations and can only be used in very narrow circumstances and very narrow situations [13] or to explore the computability of ethics in a limited domain [14]. Apart from the study on ethical framework and ethical protocol, we want to investigate the third aspect of Ethically Aligned Design on “ethical design process for HRI” which is about issues around design flow and product implementation for applying values to real products. Examples of relevant studies can be found from Marino et al. who studied the anthropometric basis for designing collaborative workplaces [15] as well as applying ISO international standards as human-centric principles in the designing phase of a human-robot collaborative environment [16]. Considering that this approach is relatively new, there is not yet a consensus about choosing which ethical design process we can follow. Hence, in this paper, we would like to examine the third aspect of the design practice of Ethically Aligned Design for human-robot interaction with a bottom-up case study of a healthcare robot design project [17]. In the meantime, we established a study group in August 2021 for a candidate project of IEEE P7000's AI ethics standards which is called “Ethical Considerations of Cognitive Robots for Enhancing Human-Efficacy.” We will also consider applying this standard to our future works for the study of Ethically Aligned Design (Figure 1).

The article "Design-Centered HRI Governance for Healthcare Robots" was published in 2022. Journal: J Healthc Eng.

Given the coexistence of humans and these “embodied” intelligent systems, we shall also consider an inside-out way of thinking when designing their sociability not from their own bodies, but from the many “social systems” in the real-world environments in which they are located. In other words, the second design-centered approach we will need to consider is called “Social System Design” [18]. In the 20th century, most robots were designed for industrial use. They worked in isolation inside factories and never had to interact with humans. However, in this century, robots will gradually enter our living environments until they fully coexist with humans. Therefore, there is a need to consider how to properly design “robot sociability.” Along this line, a micro viewpoint is to consider such design from bottom-up cases in human-robot interaction, such as Uncanny Valley or Proxemics. However, in some situations, we will need another macro viewpoint of robot sociability by using an “inside-out way.” That is to say, the subject of design is not robots but many “social systems” in the real-world environments in which these robots are located. One of the author's previous studies on Social System Design aimed to evaluate potential conflicts of traffic laws with one advanced bipedal walking humanoid robot and one human manipulated bipedal walking wheelchair inside a special zone in the downtown of Fukuoka city [19]. The other example of Social System Design was to validate potential problems of applying GDPR's informed consent obligations to the interactions with care robots via HRI experiments [20]. Next, we will consider applying Design-Centered Governance to privacy and data protection for healthcare robots through a case study.

## 3. State of the Art: Intelligent Speakers and Their Data Governance

We refer to this as “agent autonomy,” or the capability to learn and decide using machine learning and big data. In this section, we will focus on the impacts and legal concerns in regard to data protection. Although agent autonomy may raise many theoretical debates, at this moment practical cases are focused on “intelligent speakers” (like Google Home and Amazon Echo) and the risks to their privacy. One representative case is that of the Amazon Echo unit which secretly recorded a Portland couple's conversations and sent it out to their friend in Seattle [21]. Considering an intelligent speaker's strong potential for scalability with IoT devices and apps, it is worth paying attention to the data protection issues which may arise in healthcare context.

The article "Design-Centered HRI Governance for Healthcare Robots" was published in 2022. Journal: J Healthc Eng.

As of April 2019, Amazon cooperated with 6 healthcare companies to help its Echo device utilize healthcare applications. The applications they created are called “skills” which include booking medical appointments, checking on the status of a prescription, and obtaining information about instructions after being discharged from the hospital. One of the companies, Livongo Health, created an application called “Livongo Blood Sugar Lookup” which connects Alexa to a glucose monitor and allows Echo to have access to a user's blood sugar data. A year before the collaboration with the above-mentioned healthcare companies, Amazon announced plans to create software that can read medical records. Before Amazon, other companies failed in their apps development mainly because doctors take sloppy notes and use abbreviations, which are difficult for their algorithms to understand.

Amazon was able to enter the health field with Echo by making it compliant with Health Insurance Portability and Accountability Act (HIPAA). Aside from the above, Amazon also worked with the insurance provider Cigna and the healthcare provider Boston Children's Hospital. This means that Amazon Echo, as of 2019, can be used to transmit and receive sensitive personal patient data. Amazon also released a new tool called Amazon Comprehend Medical, which uses natural language processing with machine learning to analyze patient records. PillPack is an online pharmacy company that was acquired by Amazon which sends drugs to people via mail. The service was allowed to be sold in 49 states as of 2018.

From the European perspective, Amazon's Echo hardware, as well as its third party services, raises issues in regard to the General Data Protection Regulation (GDPR). Its Article 5 (1) (c) states that personal data shall be “*adequate, relevant and limited to what is necessary in relation to the purposes for which they are processed*”. This is also known as the principle of data minimization. People usually worry about their voice data being secretly collected by intelligent speakers when they had not intended to interact with the devices, especially inadequate and unnecessary voice data that is recorded and processed by devices which are on standby. However, as Jackson and Orebaugh have pointed out, before it receives a wake word, the Amazon Echo's microphone passively listens without recording or transmitting. It starts to record when the user issues the wake word and a request [22]. While this may be true, a real concern in regard to data minimization is the data controllers' tendency to keep temporal data for too long. As Roland and Conca have noted, the voice data collected for improving voice recognition should be deleted once a sufficient level of recognition is achieved [23].

The article "Design-Centered HRI Governance for Healthcare Robots" was published in 2022. Journal: J Healthc Eng.

## 4. Case Study: Healthcare Robots and the Design-Centered Approach for Data Governance

At this moment, there is no specific law to regulate agent autonomy in human-robot interactions. The closest example is GDPR's regulation on algorithmic decision making which can be found in Articles 13, 14, 15, 21, and 22. GDPR's Articles 13–15 are about the access to information and personal data, including the definition of the data subject's access right. Article 21 refers to a data subject's right to object to the processing of his or her data. In addition, the most controversial article with agent autonomy in human-robot interaction is Article 22.

GDPR's Article 22 (1), “automated individual decision making, including profiling,” states that “*the data subject shall have the right not to be subject to a decision based solely on automated processing, including profiling, which produces legal effects concerning him or her or similarly significantly affects him or her*.” In the future, there will be many services that are provided by healthcare robots based on automated decision making. It is not practicable to bind Article 22 with every piece of their decision making. The requirement for Article 22 (1) is activated when the decision (1) is based solely on automated processing, (2) produces legal effects on the individual, or (3) produces similarly significant effects on the individual. Using the Correctional Offender Management Profiling for Alternative Sanctions (COMPAS) software to access the potential recidivism risk of a criminal is an example of a decision that is based solely on automated processing which has legal effects on the individual. However, when referring to healthcare robots, there are two categories of human-robot interactions that will need to be considered by Article 22 (1). The first category pertains to algorithmic decision making in medical resource distribution and management. In the future, hospitals could potentially use big data analysis from the data pool of their patients to draw up a waiting list of patients to use their robotic surgery and healthcare services. Although this could help hospitals to manage their medical resources more efficiently, a concern is that the algorithm may miss a patient's sudden deterioration and therefore not include him or her on the priority care list. In this case, algorithmic decision making in medical resource distribution and management shall be bound by Article 22. The second category concerns algorithmic decision making in physical human-robot interactions. RIKEN's ROBEAR is a healthcare robot, classified by its makers as an “experimental nursing care robot,” designed for use in caregiving facilities. ROBEAR can perform tasks such as lifting patients. This is useful for elderly patients who might require being lifted from a bed to a wheelchair up to 40 times a day. A nursing care robot like ROBEAR equipped with agent autonomy can autonomously detect and recognize specific patients and then, based on its own judgement, decide when and how to lift the patient. A concern is that a robot like ROBEAR could accidentally cause physical injuries and bring about a tort liability claim. In this case, a patient might suffer a injury which can be classified as an issue of torts during the interaction with ROBEAR.

The article "Design-Centered HRI Governance for Healthcare Robots" was published in 2022. Journal: J Healthc Eng.

As mentioned before, we can expect an increase in cases where healthcare robots provide services with their agent autonomy. Hence, to consider under what conditions Article 22 (1) shall be applied in the two categories is a data protection issue. Generally speaking, the legal issues of the first category are similar to issues faced with current AI software. The concern to be inappropriately excluded from the priority list is a false negative problem; patients have no physical contact with robotic surgery or healthcare systems from the beginning. Hence, there would be no further dispute about whether the algorithmic decision is based solely on automated processing or not when we judge whether to apply Article 22 (1) to healthcare robots. However, in regard to algorithmic decision making in physical human-robot interactions, a dispute may arise. The risk that patients become the infringe of torts due to robots' algorithmic decision making is a false positive problem. A difficulty is to clarify the causality between the AI software's decision, the robotic hardware's execution, and the unwanted tort loss of patients.

Another question is about the legal consequences of Article 22 (1). Kaminski notes that the Article 29 Working Party guidelines clarify that Article 22 (1) is not merely a right to object to algorithmic decision making, but it includes a prohibition on it. In addition, the guidelines also hold a strict stance on narrowing the adoption of the contractual and explicit consent exceptions from Article 22 (2) (a) and (2) (c) [24]. This also generates the governance problem of maintaining a balance between regulation and innovation. It is clear that we need to draft a guideline to clarify (1) the range of medical and healthcare services which might produce legal or similarly significant effects on the individual and (2) the standard operating procedures for judging the fault of a tort action by a robot and the causality of its automated processing.

The article "Design-Centered HRI Governance for Healthcare Robots" was published in 2022. Journal: J Healthc Eng.

There is no similar legal regulation to Article 22 in the United States and Japan, even in the latest California Consumer Privacy Act (CCPA). One year before the CCPA becomes effective (California's voters approved Proposition 24 in November 2020), the California Privacy Rights Act of 2020 (CPRA) extended the current CCPA. As for agent autonomy, the CPRA will restrict the use of AI to analyzing personal data, and the new regulation is going to be effective as of January 2023.

Another key debate around Article 22 is whether it includes the right to an explanation. Kaminski points to some scholars who have argued that the right to an explanation is not included in the GDPR because it is not specifically mentioned in its text. Her argument to support the right to an explanation is based on Recital 71 which states that, “*in any case, such processing should be subject to suitable safeguards, which should include specific information to the data subject and the right to obtain human intervention, to express his or her point of view, to obtain an explanation of the decision reached after such assessment and to challenge the decision*.”

As more and more people are becoming dependent on algorithmic decision making in their daily lives, debates around the transparency of AI have increasingly focused on accountability issues. In particular, the issue of “black-box” decision making, which has been criticized as being potentially biased and unfair, has come under scrutiny. Some fear that such process could diminish people's trust in AI- and machine- driven decision making. Although the principle of transparency has been proposed as a solution in many ethical guidelines, a clear definition has yet to emerge. The purpose of asking an intelligent robot to explain its decision is that we want to avoid people's fundamental rights being infringed due to the opaque decision process of an algorithm. In other words, it is a means to realize AI transparency. However, “transparency” itself is an overused term which covers several close but not exactly identical meanings. It could refer to a fair procedure for data processing; a measure to ensure that AI is not biased, in which AI systems and related human decisions are subject to explainability; or understanding what actions the robot will take and why. Therefore, we will try to investigate the meaning of transparency.

The IEEE ethical guideline “Ethically Aligned Design (EAD)” version 2 defines AI transparency as systems “… in which it is possible to discover how and why a system made a particular decision, or in the case of a robot, acted the way it did.” Note that here the term transparency also addresses the concepts of traceability, explicability, and interpretability. While it provides a good basis for discussion, this definition still leaves many questions and hence needs to be reassessed. For example, what is the difference between “explainable AI” and “explainability” in AI transparency? There is a slight difference between traceability and transparency. The former (traceability) and verification are something developers should heed in order to ensure the safety and reliability of their system as they are fundamental to the establishment of a trustworthy relationship between a user and a machine. What we call AI transparency is more relevant to the idea that AI should be “explainable” to users and other stakeholders of robotic systems with agent autonomy in order to alleviate people's concern about unfair, biased, or other unethical decisions made by machines. When talking about explainable AI, we should understand a key difference between explainable AI and explainability. According to Miller, explainable AI means a kind of AI which explicitly tells users the decision that it made. On the other hand, explainability is closer to interpretability, which refers to a process which aims to help a human understand an outcome in a given context, as opposed to just delivering the decision [25]. In terms of robotic systems with agent autonomy, AI transparency relies more on interpretability and explainability. Fernandez et al. claim that the two terms are basically the same; the difference is mainly based on different uses of the terms AI and machine learning [26].

The article "Design-Centered HRI Governance for Healthcare Robots" was published in 2022. Journal: J Healthc Eng.

See Figure 2 [27]. According to Lipton, explainability includes both interpretability and transparency in the narrow sense. Transparency consists of three main structural factors that together form AI transparency. These are: Simulatability, Decomposability, and Algorithmic Transparency. For example, if you control the data source and remove some biased data, then you can prevent the system from giving you a biased decision. On the other hand, interpretability refers to some means to assist people to understand or discover problems inside the algorithm. It covers subtopics like Textual Descriptions, Visualizations, Local Explanations, and Examples. For example, Visualizations describes an analytical method which can be used to help engineers understand how a system operates.

To tell the difference between transparency and interpretability, we should be aware that the former asks for explainability from autonomous systems by regulating the feed data, training process, and used algorithms. Regulations on healthcare are often created in order to protect users, promote safer practices, and ensure welfare for all. It is evident by the number of data leaks and the high value associated with data today that regulation is needed to protect sensitive personal information. As for now, we already have a specific section of the GDPR regulating opaque algorithmic decision making and profiling. For agent autonomy to be widely used in various medical and healthcare applications, a possibility is that, in the future, regulating algorithms might become an independent category for regulators. However, regulating algorithms could have negative consequences, and you are regulating a tool, rather than a process. Generally, with GDPR and HIPPA, the goal is to ensure a certain process rather than a certain outcome. This is said to be done in order to make it nimbler and more adaptable to future developments. Regulating an algorithm can hurt because it is simply a tool. When one tool is unavailable, alternatives that are just as bad, or worse, could be used. Furthermore, alternatives that lead to worse health outcomes in the short run could be used as well, which is undesirable. Lastly, this could stifle innovation of an algorithm that in the long term hurts health outcomes. Bennett-Moses also notes that algorithms are not the right regulatory object. She suggests that what we need is law reform that responds to specific problems with some kind of algorithms, but not put algorithms as a category for regulation [28].

The article "Design-Centered HRI Governance for Healthcare Robots" was published in 2022. Journal: J Healthc Eng.

Except for the concern of regulation, it is unclear how transparency can function within real-world systems, especially in the case of regulating algorithmic system functions of healthcare robots with agent autonomy. In this section, we will address this issue by looking at how to apply interpretability as an alternative solution via a real case study of a sit-to-stand support healthcare robot with a Support Vector Machine (SVM) algorithm. The system (an armrest-type walker) is a prototype made by a Japanese healthcare robot maker that can provide elderly or disabled people with sit-to-stand support autonomously. In comparison to current sit-to-stand support machines which at the very least need two additional caregivers to assist the operation of the machine and to secure the users safety, the prototype can reduce manpower demand from two to one by using a machine learning algorithm (Figure 3).

As mentioned above, such prototype developments aim to enhance the efficiency of human resource distribution in care centers or hospitals. Although the manpower demand can be reduced via replacing the role of human operators by learning algorithms, one concern relates to privacy invasion confirming that a user's current state requires many sensors to collect data from the real world, including a user's biometric data. It is also unavoidable for a machine to collect sensitive data during the whole process which becomes critical for effective use of such technology. From an Ethically Aligned Design perspective, one solution for privacy protection is to control the data sources that are used by robot sensors, or to consider how to apply the principle of data minimization from GDPR and other mainstream data protection guidelines or regulations to the robot design process. Hence, designers could aim to use as few sensors as possible while retaining the same function of the healthcare robot. An alternative proposal for the compliance of data minimization principle by design from this prototype is to use the strategy of Human Center of Gravity (CoG). The basic idea is to use only pressure sensors and distance sensors from the walker to calculate a human link model, and then based on the model to get user's CoG [29].

The article "Design-Centered HRI Governance for Healthcare Robots" was published in 2022. Journal: J Healthc Eng.

In addition, the calculation of the CoG has 7 features that can be used as SVM input to classify two different states: “sitting while leaning the body” and “just sitting.” With this method, the walker will be able to decide when to activate its motor actuator to assist the patient based on user state estimation. One tricky part concerns value conflicts. Although the issue of privacy invasion can be solved using a CoG calculation, the SVM algorithm can only estimate two states from the user (“sitting” and “leaning”), and hence it contributes to the risk of system malfunction due to algorithm classification errors. The design strategy of using fewer sensors will limit the machine's perception and performance and bring with it more risk for the end user. If the system's algorithmic decision making function can judge more user states, stable and safer human-robot interaction can be promised. However, this usually means more input of real-world data points. Accordingly, a balance needs to be struck between the privacy protection and the care of the end user. Apart from potential conflicts in applying ethical values to system design processes, the black-box characteristics of the SVM learning algorithm can also raise concerns around unclear decisions. Therefore, we need to consider a design that is accountable for healthcare robots to ensure people transparency in their decision making. Our definition of design accountability of autonomous systems is that the system design has complied with Japanese Cabinet Office's Social Principles of Human-Centric AI, especially the section of Fairness, Accountability, and Transparency (FAT) [30]. Due to the limitation of user group size, this case study will skip the part of ethical compliance with algorithmic fairness or how to ensure equal treatment to people from different races, ages, or genders. As for the ethical compliance with accountability and transparency, SVM algorithm-based healthcare robots must consider the ethical design of enhancing their interpretability, since SVM itself is not a transparent model to human beings. Although the SVM algorithm can only estimate two states from the user as “sitting” and “leaning,” there is a huge safety concern when this algorithmic function is applied to physical human-robot interaction. For example, the robot might suddenly raise its armrest to scare its user if a state estimation error happened during the assistive service. To the worst case, the user might fall to the ground because of such unexpected movements from the robot. The design strategy to enhance the interpretability is to use system modeling language to connect the SVM algorithm with all of robotic hardware components (i.e., sensors, actuators, etc.) in order to show (1) how robots plan to take their actions in the real world and (2) all active hardware components at a specific time of robot malfunction. Based on the implementation of the “expression level” of human-robot interaction (a layer between the middle output of SVM algorithmic decisions and the final output of its planned actions in the real world), we can develop ethical aligned interfaces to ensure accountability and transparency in human-robot interaction [31].

The article "Design-Centered HRI Governance for Healthcare Robots" was published in 2022. Journal: J Healthc Eng.

## 5. Conclusion

Design-Centered Governance is an interdisciplinary approach to realizing the effective regulation of emerging technology. In this paper, we propose a framework based on two different design aspects: Ethically Aligned Design and Social System Design. With the advances in AI and machine learning, our society is facing the challenge of establishing a trustworthy relationship between humans and machines. A priority issue should be the realization of properly applied values in governance structures. Through a case study with a focus on the compliance of ethical principles in the design process of SVM algorithm-based healthcare robots, we also concluded that a critical challenge of applying the design-centered approach for the HRI governance will relate to keeping a balance between potential value conflicts in human-robot interaction.

## Figures and Tables

**Figure 1:** The framework of Design-Centered Governance for Autonomous Systems.

**Figure 2:** Definition of AI explainability by Lipton [27].

**Figure 3:** Human link model and the center of gravity (CoG) by Takeda et al. [29].

The article "Design-Centered HRI Governance for Healthcare Robots" was published in 2022. Journal: J Healthc Eng.

## Data Availability

This paper did not use data for an empirical study.
